# Identification of Inflammation-Related Genes and Exploration of Regulatory Mechanisms in Patients with Osteonecrosis of the Femoral Head

**DOI:** 10.1155/2022/4501186

**Published:** 2022-09-22

**Authors:** Tong Li, Cheng Huang, Jinhui Ma, Ran Ding, Qidong Zhang, Weiguo Wang

**Affiliations:** Department of Orthopedics, China-Japan Friendship Hospital, Beijing, China

## Abstract

**Background:**

Osteonecrosis of the femoral head (ONFH) is a disabling orthopedic disease, which is impacted by infiltration of immune cells. Thus, the aim of the current research was to determine the inflammation-related biomarkers in ONFH.

**Methods:**

GSE123568 dataset with control and steroid-induced osteonecrosis of the femoral head (SONFH) samples were downloaded from Gene Expression Omnibus (GEO) database. The differentially expressed genes (DEGs) were detected by limma R package and weighted gene co-expression network analysis (WGCNA) was used to explore the co-expression genes and modules. We obtained inflammation-related genes (IRGs) from the Molecular Signatures Database (MSigDB). Then, the IRGs associated with SONFH (IRGs-SONFH) were screened out and analyzed by Gene Ontology (GO) and Kyoto Encyclopedia of Genes and Genomes (KEGG) analysis. A protein-protein interaction (PPI) network was established using the Search Tool for the Retrieval of Interacting Genes/Proteins (STRING) database, and hub genes were identified by the MCODE algorithm. Based on the hub genes, we constructed a lncRNA-miRNA-mRNA network.

**Results:**

We identified 535 DEGs between control and SONFH samples. The WGCNA clearly indicated that the brown module was most significantly associated with SONFH. We identified 25 IRGs-SONFH through WGCNA module genes, DEGs and IRGs. A total of 4 hub genes (CD14, CYBB, NOD2, and TLR1) were identified by Cytoscape. Receiver operating characteristic (ROC) curve analysis determined that the expressions of the four genes could distinguish SONFH from controls as evidenced by the area under the curve (AUC) greater than 0.7. Finally, we constructed a competitive endogenous RNA (ceRNA) network which included 67 lncRNAs, 1 miRNA (hsa-miR-320a), and 1 mRNA (NOD2).

**Conclusions:**

Our study identified 4 hub genes as potential inflammation-related biomarkers of SONFH. Moreover, we proposed a ceRNA network of lncRNAs targeting hsa-miR-320a, hsa-miR-320a, and NOD2 as a potential RNA regulatory pathway that controls disease progression in ONFH.

## 1. Background

Osteonecrosis of the femoral head (ONFH) is characterized by the death of bone due to the circulatory disruption of the femoral head with traumatic or nontraumatic factors [1]. As a large range of diseases requires steroid usage, steroid-induced osteonecrosis of the femoral head (SONFH) accounts for a large proportion of ONFH [2]. There are approximately 8.12 million nontraumatic ONFH cases in the population aged 15 years and over in China, among which SONFH counts for 47.4% [3]. Association Research Circulation Osseous (ARCO) classification system [4] was developed for accurate staging, which is essential for successful treatment. As the early symptoms of ONFH are not obvious, patients are often diagnosed at the advanced stage (ARCO stage III-IV). Therefore, novel diagnostic biomarkers and therapeutic targets are urgently needed to provide for intervention and treatment of SONFH patients.

In previous studies, inflammation has been shown to play an indispensable role in the development and progression of SONFH. Li et al. identified 8 candidate serum biomarkers of SONFH and found they were significantly involved in immune regulation and inflammation [5]. Real-time imaging probes showed the accumulation of elevated neutrophils and macrophages in the tissue of osteonecrosis in a mouse model [6]. Necrotic bone stimulated macrophage-inflammatory response through activation of a pattern recognition receptor (PRR) Toll-like receptor 4 (TLR4) and upregulation of the downstream transcription factors, including Nuclear factor-kappa B (NF-*κ*B) and monocyte chemotactic protein 1 (MCP-1), for inflammatory proteins [7, 8]. In other studies, the levels of pro-inflammatory cytokines interleukin (IL)-9, IL-17, IL-23, and IL-33 produced by T cells have been reported to be associated with ONFH [9–12]. In addition, the activation of specific B cells and elevated levels of serum Tumor necrosis factor *α* (TNF-*α*) were associated with the development of ONFH [13]. Moreover, neutrophil granulocyte levels and percentage of neutrophil granulocytes were related to ONFH [14].

Bioinformatics has been used to identify hub genes, interaction networks, and pathways of SONFH to improve diagnosis and treatment. Early studies identified biomarkers of SONFH based on weighted gene co-expression network analysis (WCGNA) and differentially expressed genes (DEGs) screening and further revealed their correlation with immune infiltration [15, 16]. Competitive endogenous RNA (ceRNA) networks can reveal potential mechanisms of disease in transcriptional regulatory networks, while no study has been conducted to analyze it in osteonecrosis.

In the present study, we proposed to identify novel inflammation-related biomarkers and evaluate its diagnostic value in SONFH on the basis of GSE123568 dataset. The DEGs screening, WCGNA, and inflammation-related gene (IRG) expression were used to identify the gene network signature and IRGs associated with SONFH (IRGs-SONFH). Then, the IRGs-SONFH was analyzed by Gene Ontology (GO) and Kyoto Encyclopedia of Genes and Genomes (KEGG) analysis, and the protein-protein interaction (PPI) was constructed. Subsequently, 4 hub genes were screened out and verified by quantitative reverse transcription polymerase chain reaction (qRT-PCR). Finally, we constructed a ceRNA network to get a deep understanding of the pathogenesis of ONFH on the basis of the predicted results of microRNAs (miRNAs) and long non-coding RNAs (lncRNAs). The research process of this study is shown in Figure 1.

## 2. Methods

### 2.1. Data Source

Microarray RNA expression dataset of GSE123568 was downloaded from the Gene Expression Omnibus (GEO) database (https://www.ncbi.nlm.nih.gov/geo/). The GSE123568 dataset was generated from samples of peripheral serum in 30 SONFH patients (steroid-induced femoral head necrosis samples) and 10 non-SONFH patients as controls. The dataset was based on the platform GPL15207 ([PrimeView] Affymetrix Human Gene Expression Array). The array data for GSE89587 included the miRNA expression profiles of 10 ONFH patients (traumatic femoral head necrosis samples) and 10 controls to construct a ceRNA network. 200 IRGs were obtained from the HALLMARK_INFLAMMATORY_RESPONSE gene set in the Molecular Signature Database (MSigDB) (https://www.broadinstitute.org/msigdb) [17].

### 2.2. Identification of DEGs

The limma, a package in the R language, was used to identify DEGs with the cut-off point of adjusted *p*-value (false discovery rate) <0.05 and |Log_2_fold change| >1. Heatmap and volcano plots of DEGs from the databases were constructed with Pheatmap and ggplot2 R packages.

### 2.3. Construction of Weighted Gene Co-Expression Networks

The R package WGCNA [18] was used to analyze the gene co-expression network of the GSE123568 dataset. First, the samples were clustered and the outliers were removed. Second, to construct a scale-free network, the soft threshold of *β* =18 was chosen with the function pickSoftThreshold. Based on the selected soft threshold, the adjacency matrix was converted to topological overlap matrix for constructing the network, and the gene dendrogram and module color were established by utilizing the degree of dissimilarity. Then, the correlations between modules and SONFH were calculated using the WGCNA package. Therefore, modules with high correlation coefficient were considered candidates relevant to SONFH and were selected for subsequent analysis. The intersection of DEGs, genes in key modules, and IRGs were carried out using the “VennDiagram” R package and were defined as IRGs-SONFH, which were used for subsequent analysis.

### 2.4. KEGG and GO Enrichment Analysis

Functional annotation of IRGs-SONFH was presented with the R package “clusterProfiler” [19], containing GO and KEGG pathway analysis. GO terms were comprised of the biological process (BP), cellular component (CC), and molecular function (MF) [20] and were used to identify the biological properties of genes and gene sets in all organisms. The KEGG enrichment analysis was performed to obtain the associated enrichment pathways. Adjusted *p*-value <0.05 was considered statistically significant.

### 2.5. Construction of PPI Network

The Search Tool for the Retrieval of Interacting Genes/Proteins (STRING) database (https://cn.string-db.org/cgi/input?sessionId=bbRkt711IuEL&input_page_active_form=multiple_identifiers) [21] was used to construct a PPI network of the above genes. Next, we downloaded the interaction information and optimized the PPI network with Cytoscape software (https://www.cytoscape.org) [22] for better visualization. The MCODE plug-in in Cytoscape was used to identify significant gene clusters and obtain hub genes. The hub genes were evaluated using the geometric mean of semantic similarities in CCs and MFs by applying the “GOSemSim” package in R software [23]. Corrplot package was used to analyze the correlation of hub genes.

### 2.6. qRT-PCR

The serum samples of 24 patients with femoral neck fracture and 24 patients with SONFH were acquired for qRT-PCR to verify the predictive analysis results. Total RNA was extracted from the serum samples using TRIzol, and then, its concentration and purity were assessed by nanodrop. RNA samples from total RNA were reverse-transcribed to cDNA, and qRT-PCR was performed using the SuperScript III RT (ABI-Invitrogen, 11752050). *β*-Actin was used as an internal normalization standard. The 2^−*ΔΔ*Ct^ method was utilized to determine the relative expression of each selected gene between SONFH and controls. Sequences of primers used in the study are shown in Table 1. Student's *t*-test was used to compare the differences between the 2 groups.

### 2.7. The Receiver Operating Characteristic (ROC) Curve Analysis and Expression Analysis

In the GSE123568 dataset, 30 SONFH samples and 10 control samples were utilized to plot ROC curves, from which we obtained their area under the ROC curves (AUC) through the “pROC” package. ROC curve is a helpful tool to evaluate the efficiency of gene diagnosis. The hub genes with AUC >0.7 were deemed useful for disease diagnosis.

Expression levels of hub genes between SONFH and normal samples were shown using boxplots. The boxplots of hub gene expression were drawn using the “ggplot2” in R package.

### 2.8. Correlation Analysis between Hub Genes and Infiltrated Immune Cells

Immune infiltration analysis was performed by using the ssGSEA algorithm. Correlation analysis between crucial genes and 28 immune cells was calculated via the Spearman method, and the results were visualized. Correlation analysis was conducted to determine the relationship between hub genes and differential immune cells.

### 2.9. Small-Molecule Drug Prediction and Gene Set Enrich Analysis (GSEA)

The latent drugs for hub genes were predicted through the Drug-Gene Interaction Database (DGIdb) (https://dgidb.org/search_interactions) [24]. We used the R package “clusterprofiler” to conduct GSEA on hub genes. The chosen reference gene set was downloaded from the MSigDB. A *p*-value < 0.05 was considered statistically significant.

### 2.10. Prediction of Networks Mutually Regulated by miRNAs and Transcription Factors (TFs)

The upstream TFs and miRNAs were predicted using the miRNet database (https://www.mirnet.ca) [25]. Subsequently, the results were visualized using Cytoscape software.

### 2.11. CeRNA Network Construction

To predict the regulatory relationship among mRNAs, lncRNAs, and miRNAs, lncRNAs were predicted using miRNet. Briefly, differentially expressed miRNAs (DEmiRNAs) in GSE89587 with the threshold criterion of adjusted *p* value (false discovery rate) <0.05 and |Log_2_fold change| =0 were screened using the limma package of the R software program. Then, they were intersected with the miRNAs predicted by the hub genes to get the final target miRNAs. Target lncRNAs matched by target miRNAs were retrieved from the miRNet database. The ceRNA regulatory network of lncRNA-miRNA-mRNA was visualized using Cytoscape software.

## 3. Results

### 3.1. Identification of DEGs

In our study, 535 DEGs were identified between SONFH samples and control samples. Among them, 299 were upregulated and 236 were downregulated (SONFH vs. control). The volcano plot and heat map of gene expression are shown in Figures 2(a) and 2(b).

### 3.2. Construction of Co-Expression Networks

The sample clustering tree indicated that there was no abnormal sample (Figures 3(a) and 3(b)). After calculation, the best soft-thresholding power was set at 18 (Figure 3(c)). Finally, each module was assigned a color, and a total of 9 modules in GSE123568 (Figure 3(d)) were identified in this study. Furthermore, the result of the module-feature relationship revealed that the brown module had the highest correlation with SONFH (cor =0.68, *p* = 1e−05, Figure 3(e)). Thus, 850 genes in the brown module were selected for further exploration.

### 3.3. Identification of IRGs-SONFH and Functional Enrichment Analysis

Then, we took the intersection of DEGs, genes in key modules, and IRGs and identified 25 IRGs-SONFH (Figure 4(a)). To explore the function of 25 IRGs-SONFH in SONFH, the GO terms are shown in Figure 3. In BP analysis (Figure 4(b)), IRGs-SONFH mainly participated in response to molecules of bacterial origin, neutrophil activation, response to lipopolysaccharide, cellular response to biotic stimulus, and cellular response to molecule of bacterial origin. In CC analysis (Figure 4(c)), IRGs-SONFH significantly participated in the membrane microdomain, membrane raft, secretory granule membrane, endocytic vesicle, and phagocytic vesicle. MF analysis showed that IRGs-SONFH significantly participated in amide binding, peptide binding, immune receptor activity, pattern recognition receptor activity, and lipopolysaccharide binding (Figure 4(d)). KEGG analysis was performed to explore the pathways of these 25 IRGs-SONFH. The KEGG terms of IRGs-SONFH are shown in Figure 4(e). As shown, these IRGs-SONFH were mainly enriched in lipid and atherosclerosis, tuberculosis, neutrophil extracellular trap formation, TLR signaling pathway, and legionellosis.

### 3.4. Identification of Hub Genes

The PPI network between IRGs-SONFH was established using the STRING database; the interactions of 25 IRGs-SONFH are displayed in Figure 5(a). 4 hub genes (CD14, CYBB, NOD2, and TLR1) were identified by MCODE plug-in Cytoscape (Figure 5(b)).

### 3.5. The Correlation Analysis between Hub Genes and the Functional Similarity Analysis of Hub Genes

The correlation between these 4 hub genes was investigated using the corrplot package; CD14 and TLR1 had the strongest correlation (*r* =0.85) (Figure 5(c)). We analyzed the functional similarity of these hub genes by the “GOSemSim” package in R. The results showed that 3 hub genes, including CD14, NOD2, and TLR1 (similarity score > 0.5), had higher functional similarity (Figure 5(d)).

### 3.6. Validation and Efficacy Evaluation of Hub Genes

We explored the expressions of these genes between SONFH and control samples in GSE123568 and found that those genes exhibited higher expression levels in SONFH (Figure 6(a)). In addition, the relative expressions of the above four hub genes were investigated by qRT-PCR. As shown in Figures 6(c)–6(f), the relative expressions of CD14, CYBB, NOD2, and TLR1 were also significantly increased in the peripheral blood of SONFH patients compared to controls. Furthermore, we executed a ROC curve analysis to calculate their sensitivity and specificity for the diagnosis of SONFH (Figure 6(b)). The AUC values of CD14, CYBB, NOD2, and TLR1 were 0.847, 0.753, 0.767, and 0.847, respectively, demonstrating that these genes have high sensitivity and specificity for SONFH diagnosis.

### 3.7. Correlation Analysis of Hub Genes and Immune Cells

To further understand the role of these genes in immune infiltration, we used Spearman's correlation analysis to determine whether these hub genes were related to immune cell infiltration. Correlation analysis showed that 4 hub genes including CD14, CYBB, NOD2, and TLR1 had significantly positive relationship with type 1 T helper cell, T follicular helper cell, regulatory T cell, plasmacytoid dendritic cell, neutrophil, natural killer T cell, natural killer cell, monocyte, memory B cell, myeloid-derived suppressor cell, mast cell, macrophage, immature dendritic cell, immature B cell, gamma delta T cell, eosinophil, effector memory CD8 T cell, effector memory CD4 T cell, central memory CD4 T cell, central memory CD8 T cell, and activated dendritic cell (Figure 7).

### 3.8. GSEA

The function of our hub genes was explored via GSEA. Genes in the high-expression cohorts of CD14 and TLR1were all highly enriched in leishmania infection, Toll-like receptor signaling pathways, and Fc gamma R-mediated phagocytosis (Figures 8(a) and 8(d)). Genes in the high-expression cohorts of CYBB and NOD2 were all highly enriched in spliceosome, lysosome, and B-cell receptor signaling pathways (Figures 8(b) and 8(c)). Genes in the low-expression cohorts of CD14, CYBB, NOD2, and TLR1 were all highly enriched in olfactory transduction, linoleic acid metabolism, and basal cell carcinoma (Figure 8). After considering the results of GSEA, we concluded that these four genes might be highly correlated with immune and inflammation.

### 3.9. Drug-Gene Networks

A total of 17 potential drugs for treating SONFH patients were identified when the drug-gene interactions were explored using DGIdb (Table 2). Additionally, drug-gene networks were constructed by Cytoscape (Figure 9(a)). However, we did not find any small-molecule drugs that could target TLR1 in this database.

### 3.10. Prediction of Key miRNAs and TF

The miRNA and TFs regulatory network of 4 hub genes was constructed using miRNet. As illustrated in Figure 9(b), the interaction network consisted of 4 hub genes and 59 miRNAs. Specifically, 9 miRNAs (i.e., hsa-mir-335-5p, hsa-mir-100-5p, hsa-mir-3687) targeting CD14, 28 miRNAs (i.e., hsa-mir-6826-3p, hsa-mir-6845-3p, hsa-mir-6859-3p) targeting CYBB, 12 miRNAs (i.e., hsa-mir-215-5p, hsa-mir-122-5p, hsa-mir-320a) targeting NOD2, and 15 miRNAs (i.e., hsa-mir-34a-5p, hsa-mir-3662, hsa-mir-4511) targeting TLR1. The interaction network consisted of 4 hub genes and 30 TFs. We found that 12 TFs (i.e., CEBPB, FOS, JUN) could regulate CD14. 8 TFs (i.e., NFIC, NFYA, YY1) could regulate CYBB. 11 TFs (i.e., MAX, USF1, USF2) could regulate NOD2. 8 TFs (i.e., MEF2A, HINFP, TP63) could regulate TLR1.

### 3.11. CeRNA Regulatory Network Construction

To elucidate the potential molecular mechanism of lncRNAs in SONFH, we constructed a lncRNA-miRNA-mRNA interaction network. Briefly, 20 DEmiRNAs with the threshold criterion of adjusted *p*-value < 0.05 and |Log_2_fold change|=0 were screened by GSE89587. 1 miRNA (hsa-miR-320a) was obtained by taking the intersection of 64 miRNAs predicted by the hub genes above and 20 DEmiRNAs. We used the database miRNet to predict the lncRNAs that interacted with the selected miRNAs (hsa-miR-320a). Finally, we obtained a ceRNA network which included 67 lncRNAs, 1 miRNA (hsa-miR-320a), and 1 mRNA (NOD2) (Figure 9(c)).

## 4. Discussion

ONFH is a progressive disease with necrosis of the osteocyte and bone marrow as a result of intramedullary microvascular lesions and interruption of blood supply of the femoral head. In patients with end-stage ONFH, collapse of the femoral head can lead to dysfunction of the hip joint, ultimately affecting the quality of life. Hence, novel biomarkers for early diagnosis and individualized treatment are urgently needed. Multiple biological processes, including circulation, steroid metabolism, immunity, and bone formation, were involved in the development of ONFH [26]. Although existing theories have pointed to the role of inflammation in the pathogenesis of SONFH [15], the molecular mechanism contributing to disease onset remains unclear. In addition, few studies have systematically screened the biomarkers related to inflammation and their value for assessing the process of SONFH.

In this study, a total of 535 DEGs were identified in the SONFH and control samples. In addition, 9 co-expression modules were obtained by WGCNA analysis. Among them, the brown module with a total of 850 genes was the most relevant to SONFH. Moreover, 200 IRGs were identified. We obtained 25 candidate genes for hub genes by taking the intersection of the above three gene lists. Bioinformatics databases, including GO and KEGG, are widely used in gene classification and signaling pathway analysis. As demonstrated from GO enrichment results, the candidate genes showed a major relationship with the response to the molecule of neutrophil activation, PRR signaling pathway, and TLR2 signaling pathway. In addition, KEGG pathways were enriched in neutrophil extracellular trap formation, TLR signaling pathway, NF-*κ*B signaling pathway, and NOD-like receptor signaling pathway. Although SONFH is not an inflammatory disease, the enrichment results suggest that inflammation may play a critical role in its pathophysiological mechanism.

Through PPI network, we identified 4 hub genes, namely, CD14, CYBB, NOD2, and TLR1. As shown by the ROC curve, they had high sensitivity and specificity for SONFH and could be used as biomarkers. Furthermore, qRT-PCR showed that the relative expression of CD14, CYBB, NOD2, and TLR1 in the peripheral blood samples of SONFH was increased compared with normal group. Finally, we constructed a ceRNA network to clarify the pathogenesis of ONFH from the transcriptomic level.

The protein encoded by CD14 is a surface antigen which is preferentially expressed on monocytes and macrophages. Generally, macrophages are known as a critical role in the innate immune response and they can polarize into pro-inflammatory (M1) or anti-inflammatory (M2) phenotypes depending on the microenvironment [27]. The repolarization of macrophages from the M1 phenotype to M2 phenotype could promote the survival of osteocytes and decrease inflammatory cytokines, which was effective in the alleviation of SONFH [28]. Early study has shown that CD14+ macrophages increased in the fibrovascular repair tissue during the induction of ONFH [7]. Consistent with the present study, we found that CD14 expression was upregulated in SONFH patients and the ROC curve showed that CD14 had a high diagnostic value (AUC =0.847).

CYBB is a transmembrane protein of the microbicidal oxidase system of phagocytes [29]. CYBB deficiency can lead to the disorder of reactive oxygen species (ROS) production, resulting in the disability of phagocytes to kill most pathogens, which is associated with the rare immune deficiency disorder, chronic granulomatous disease [30]. However, uncontrolled neutrophil ROS production can lead to persistent vascular inflammation reactions contributing to some inflammatory diseases [31]. Moreover, the impaired blood vessels caused by dysregulation of bone endothelial cells are one of the most convincing mechanisms of SONFH [32]. Therefore, the vascular inflammation caused by high expression of CYBB may be related to SONFH. In the current study, we found that CYBB expression was upregulated in SONFH patients and it may be a diagnostic biomarker for SONFH (AUC =0.753).

NOD2 is one of PRRs of the NOD-like receptor (NLR) family that sense conserved motifs in bacterial peptidoglycan and activate intracellular signaling pathways that drive pro-inflammatory and antimicrobial responses [33]. NOD2 regulates multiple pathways involved in a variety of inflammatory responses via the activation of NF-*κ*B, MAPK, and type I interferons (IFN) [34, 35]. NOD2 also interplays with TLRs during systemic bacterial infection to enhance immune response and promote immune responses after toleration by TLR ligands [36]. Furthermore, the activation of TLR4/NF-*κ*B pathway results in the gene expression of molecules responding to inflammatory cytokine responses in macrophages, which may contribute to SONFH [37, 38]. Therefore, combined with the results of the ROC curve (AUC =0.767), we hypothesize that NOD2 may be an effective biomarker for the diagnosis of SONFH.

TLR1 is a member of the TLR family, which is responsible for the recognition of pathogen-associated molecular patterns (PAMPs) and induction of inflammatory immune responses [39]. The formation of TLR1-TLR2 heterodimer brings the intracellular Toll/interleukin 1 receptor (TIR) domains into close proximity and initiates signaling [40]. MyD88, an intracellular TIR-containing adaptor used by TLR1, interacts with interleukin-1 receptor-associated kinases (IRAKs) and eventually leads to the activation of NF-*κ*B and IFN-regulatory factors (IRFs) to elicit anti-pathogen responses and inflammation [41]. Our study showed that the expression of TLR1 increased in SONFH patients and TLR1 had a high diagnostic value according to the ROC curve (AUC =0.847). Therefore, we believe that TLR1 is a new and effective biomarker for the diagnosis of SONFH.

Furthermore, miRNAs and TFs targeting CD14, CYBB, NOD2, and TLR1 were predicted and a total of 20 differentially expressed miRNAs were identified in patients with osteonecrosis and controls. Among the 20 differentially expressed miRNAs, hsa-miR-320a was found as a regulatory miRNA of NOD2. Consequently, lncRNAs targeting hsa-miR-320a were searched from the database and a ceRNA network of 67 lncRNAs targeting hsa-miR-320a, hsa-miR-320a, and NOD2 was constructed. In early bioinformatics researches, hsa-miR-320a has been identified as diagnostic biomarker of atherogenesis [42], multiple sclerosis [43], gastric cancer [44], and metabolic syndrome [45]. Our study indicated that hsa-miR-320a was a key regulator of NOD2 associated with inflammation contributing to the progression of osteonecrosis.

This study had several limitations. The sample size for analysis and validation was relatively small. Moreover, most SONFH cases have other comorbidities which have been treated with glucocorticoids, and the different primary diseases may influence our results. Therefore, future studies need to increase the sample size and control the effects of primary disease to further confirm our results.

## 5. Conclusions

This study identified and validated 4 hub genes, CD14, CYBB, NOD2, and TLR1, as potential inflammation-related biomarkers of SONFH, and provided clues to the mechanism of disease development of SONFH at the transcriptome level. Moreover, we proposed a ceRNA network of lncRNAs targeting hsa-miR-320a, hsa-miR-320a, and NOD2 as a potential RNA regulatory pathway that controls disease progression in ONFH.

## Figures and Tables

**Figure 1:** Flowchart of data processing. GEO: Gene Expression Omnibus; DEG: differentially expressed gene; WCGNA: weighted gene co-expression network analysis; SONFH: steroid-induced osteonecrosis of the femoral head; IRG: inflammation-related gene; GO: Gene Ontology; KEGG: Kyoto Encyclopedia of Genes and Genomes; PPI: protein-protein interaction; ROC: receiver operating characteristic; qRT-PCR: quantitative reverse transcription polymerase chain reaction; GSEA: Gene Set Enrich Analysis; miRNA: microRNA; TF: transcription factor; ceRNA: competitive endogenous RNA.

**Figure 2:** The volcano plot and heat map of gene expression. (a) Volcano plot of GSE123568, mRNAs. (b) Heat map analysis of GSE123568, mRNAs. Differentially expressed mRNA molecules were screened under the cut-off criteria adjusted *p* value (false discovery rate) <0.05 and |Log_2_fold change|>1. The 10 most significantly upregulated genes and the most significantly downregulated genes were selected for heat map visualization.

**Figure 3:** The WGCNA of GSE123568. (a) Sample clustering to detect outliers. (b) Sample dendrogram and trait heat map. (c) Analysis of the scale-free fit index for various soft-thresholding powers and analysis of the mean connectivity of various soft-thresholding powers. (d) The cluster dendrogram of genes. (e) Module-trait relationships.

**Figure 4:** Analysis results of IRGs-SONFH in the GO and KEGG. (a) A total of 25 IRGs-SONFH were identified by the intersection of DEGs, genes in key modules, and IRGs. (b) Results of GO biological process analysis. (c) Results of GO cellular component analysis. (d) Results of GO molecular function analysis. (e) Results of KEGG pathway analysis.

**Figure 5:** Identification, correlation analysis, and functional similarity analysis of hub genes. (a) The PPI network between 25 IRGs-SONFH. Each node represents a protein, while each edge represents one protein-protein association. (b) A total of 4 hub genes were identified by MCODE plug-in Cytoscape. (c) Results of correlation analysis between the 4 hub genes. (d) Results of functional similarity analysis of the 4 hub genes.

**Figure 6:** Validation and efficacy evaluation of the 4 hub genes. (a) The 4 hub genes exhibited higher expression levels in SONFH than controls in GSE123568. (b) ROC curves of the 4 hub genes showed high sensitivity and specificity for SONFH diagnosis. (c–f) Results qRT-PCR showed that the relative expressions of CD14, CYBB, NOD2, and TLR1 were also significantly increased in peripheral blood of SONFH patients compared to controls.

**Figure 7:** Correlation analysis of the hub genes and immune cells. The color of the spots represents the *p* value, while the size represents the gene number.

**Figure 8:** GESA results of the 4 hub genes. (a) CD14; (b) CYBB; (c) NOD2; (d) TLR1.

**Figure 9:** Drug-gene networks and ceRNA network. (a) Drug-gene networks constructed by Cytoscape. (b) Interaction network consisted of 4 hub genes, 59 miRNAs, and 30 TFs. (c) A ceRNA network which included 67 lncRNAs, 1 miRNA (hsa-miR-320a), and 1 mRNA (NOD2).

**Table 1:** Primer information.

Target name		Primer
*β*-Actin	F	GACAGGATGCAGAAGGAGATTACT
	R	TGATCCACATCTGCTGGAAGGT
NOD2	F	TTGCCTAGTTCTGGAAGGCTG
	R	CCTCTTCCCCCATCAAAGCC
CYBB	F	GCAGGAAAGGAACAATGCCG
	R	CATTATCCCAGTTGGGCCGT
TLR1	F	GCCACCCTACTGTGAACCTC
	R	ATGAGCAATTGGCAGCACAC
CD14	F	ACAGGTGCCTAAAGGACTGC
	R	GATTCCCGTCCAGTGTCAGG

**Table 2:** Potential drugs for treating SONFH.

Gene	Drug	Sources	Pmids
NOD2	CHEMBL1456848	DTC	
NOD2	CHEMBL585502	DTC	
NOD2	MIFAMURTIDE	ChemblInteractions	20596505|21226638
NOD2	INARIGIVIR SOPROXIL	TTD	
NOD2	CHEMBL599890	DTC	
NOD2	CHEMBL578944	DTC	
NOD2	CHEMBL577660	DTC	
NOD2	MURABUTIDE	DTC	22716113
NOD2	TACROLIMUS	PharmGKB	23175667
NOD2	CHEMBL590706	DTC	
NOD2	CHEMBL1351908	DTC	
NOD2	CYCLOVALONE	DTC	
CYBB	APIGENIN	DTC	23786520
CYBB	CHRYSIN	DTC	23786520
CYBB	LUTEOLIN	DTC	23786520
CD14	IC14	TdgClinicalTrial|ChemblInteractions|TTD	
CD14	LOVASTATIN	NCI	7506029

## Data Availability

The datasets generated and analyzed during the current study are available in the GEO, MSigDB, STRING, DGIdb, and miRNet databases. GEO (https://www.ncbi.nlm.nih.gov/geo/); MSigDB (https://www.broadinstitute.org/msigdb); STRING (https://string-db.org); DGIdb (https://www.dgidb.org); miRNet (https://www.mirnet.ca).

## Abbreviations

ONFH: Osteonecrosis of the femoral head
SONFH: Steroid-induced osteonecrosis of the femoral head
ARCO: Association Research Circulation Osseous
PRR: Pattern recognition receptor
TLR4: Toll-like receptor 4
NF-*κ*B: Nuclear factor-kappa B
MCP-1: Monocyte chemotactic protein 1
IL: Interleukin
TNF-*α*: Tumor necrosis factor *α*
WCGNA: Weighted gene co-expression network analysis
DEG: Differentially expressed gene
ceRNA: Competitive endogenous RNA
IRG: Inflammation-related gene
GO: Gene Ontology
KEGG: Kyoto Encyclopedia of Genes and Genomes
qRT-PCR: Quantitative reverse transcription polymerase chain reaction
miRNA: MicroRNA
lncRNA: Long non-coding RNA
GEO: Gene Expression Omnibus
MSigDB: Molecular Signature Database
BP: Biological process
CC: Cellular component
MF: Molecular function
PPI: Protein-protein interaction
STRING: Search Tool for the Retrieval of Interacting Genes/Proteins
ROC: Receiver operating characteristic
AUC: Area under curve
DGIdb: Drug-gene interaction database
GSEA: Gene set enrich analysis
TF: Transcription factor
DEmiRNA: Differentially expressed miRNA
NLR: NOD-like receptor
IFN: Interferons
ROS: Reactive oxygen species
PAMP: Pathogen-associated molecular pattern
TIR: Toll/interleukin 1 receptor
IRAK: Interleukin-1 receptor-associated kinase
IRF: IFN-regulatory factor.
